# Performance Evaluation of Machine Learning Algorithm for Classification of Unintended Pregnancy among Married Women in Bangladesh

**DOI:** 10.1155/2022/1460908

**Published:** 2022-05-28

**Authors:** Md. Ismail Hossain, Md. Jakaria Habib, Ahmed Abdus Saleh Saleheen, Md. Kamruzzaman, Azizur Rahman, Sutopa Roy, Md. Amit Hasan, Iqramul Haq, Md. Injamul Haq Methun, Md. Iqbal Hossain Nayan, Md. Rukonozzaman Rukon

**Affiliations:** ^1^Department of Statistics, Jagannath University, Dhaka 1100, Bangladesh; ^2^Department of Statistics, Jahangirnagar University, Savar, Dhaka, Bangladesh; ^3^Department of Agricultural Statistics, Sher-e-Bangla Agricultural University, Dhaka 1207, Bangladesh; ^4^Statistics Discipline, Tejgaon College, Dhaka 1215, Bangladesh; ^5^Quality Services and Compliance, Square Pharmaceutical Limited, Dhaka, Bangladesh

## Abstract

Intended pregnancy is one of the significant indicators of women's well-being. Globally, 74 million women become pregnant every year without planning. Unintended pregnancies account for 28% of all pregnancies among married women in Bangladesh. This study aimed to investigate the performance of six different machine learning (ML) algorithms applied to predict unintended pregnancies among married women in Bangladesh. From BDHS 2017-18, only 1129 pregnant women aged 15–49 were eligible for this study. An independent *χ*^2^ test had performed before we considered six popular ML algorithms, such as logistic regression (LR), random forest (RF), support vector machine (SVM), k-nearest neighbor (KNN), naïve Bayes (NB), and elastic net regression (ENR) to predict the unintended pregnancy. Accuracy, sensitivity, specificity, Cohen's Kappa statistic, and area under curve (AUC) value were used as model evaluation. The bivariate analysis result showed that women aged 30–49 years, poor, not educated, and living in male-headed households had a higher percentage of unintended pregnancy. We found various performance parameters for the classification of unintended pregnancy: LR accuracy = 79.29%, LR AUC = 72.12%; RF accuracy = 77.81%, RF AUC = 72.17%; SVM accuracy = 76.92%, SVM AUC = 70.90%; KNN accuracy = 77.22%, KNN AUC = 70.27%; NB accuracy = 78%, NB AUC = 73.06%; and ENR accuracy = 77.51%, ENR AUC = 74.67%. Based on the AUC value, we can conclude that of all the ML algorithms we investigated, the ENR algorithm provides the most accurate classification for predicting unwanted pregnancy among Bangladeshi women. Our findings contribute to a better understanding of how to categorize pregnancy intentions among Bangladeshi women. As a result, the government can initiate an effective campaign to raise contraception awareness.

## 1. Introduction

Unintended pregnancy, also known as unwanted pregnancy, is a global public health issue in low- and middle-income countries/regions [1]. On a global scale, 74 million women become pregnant every year without planning [2]. Although the unexpected pregnancy rate has decreased over time, the rate has not decreased much in developing countries [3]. In Asia, there are approximately 53.8 million unplanned pregnancies each year. In Africa, 8 out of 100 women have unplanned pregnancies, and Eastern Africa has the highest rate [4].

Unintended pregnancy can cause maternal death and morbidity due to pregnancy-related complications (such as unsafe abortions and unplanned births) [5]. In developing countries, 40% of pregnancies are unexpected, resulting in 25 million unsafe abortions and 47,000 maternal deaths each year [2].

Previous studies based on the Demographic Health Survey's (DHS's) data have shown that unplanned pregnancies among married women are still a global health problem. According to a recent DHS survey, the unexpected pregnancy rate in Ethiopia is 28% [6]. Another study of a Ugandan woman who is currently married found that 37% of pregnancies were unplanned [7]. Research based on data from six South Asian countries shows that about 28% of married women in Bangladesh have unintended pregnancies. Also, in Bangladesh's neighboring country (India), unwanted pregnancies are 12% [8].

Planning to become pregnant may be the best indicator of women's well-being [9]. The causes of unwanted pregnancy are many and complex. Failure to use contraceptives is widely considered the main cause of unintended pregnancy [10]. The previous study found that different variables are significantly related to unwanted pregnancy, such as maternal age, maternal education, wealth index, maternal age at first marriage, and birth [7, 8].

Through proper family planning, diagnosis, and intervention measures, unnecessary pregnancy and miscarriage can be reduced. Various statistical methods (Binary Logistic Regression analysis) have been applied to determine the significant indicators of unintended pregnancy in married women. The main goal of the diagnostic procedure is to correctly predict pregnancy intentions. Machine learning is a scientific method that can build models for prediction purposes. Various recent studies in the literature indicate that machine learning, as well as deep learning, can significantly improve predictive performance [11–13]. In recent times, researchers have used various machine learning algorithms to study prediction performance [11]. All in all, machine learning is now being used everywhere in the research sector. Nowadays, machine learning is very popular in health-related fields [14–18].

However, not many studies have considered machine learning techniques to develop prediction models for unwanted pregnancies among married women. Therefore, in this study, various well-known machine learning algorithms have been applied to predict unintended pregnancies among married women in Bangladesh.

## 2. Materials and Methods

### 2.1. Data Source

This study used nationally representative secondary data, named Bangladesh Demographic and Health Survey (BDHS), 2017-18. The authority designed the survey to collect household data to monitor and evaluate children and mothers' health status, including nutrition, causes of death, newborn care, empowerment of women, and more. The United States Agency for International Development (USAID) in Bangladesh provided financial support for this investigation. The data is publicly available for research.

### 2.2. Sampling Design and Sample Size

The Demographic Health Survey Authority used a two-step stratified sampling procedure in the 2017-18 Bangladesh Demographic Health Survey (BDHS). The data comes from eight divisions: Barisal, Chattogram, Dhaka, Khulna, Mymensingh, Rajshahi, Rangpur, and Sylhet. The survey used the list of the enumerated area (EA) of the population and housing census of Bangladesh in 2011 provided by the Bangladesh Statistics Office (BBS). In the first stage, 675 EAs were selected, including 250 EAs in urban areas and 425 EAs in rural areas. In the survey, 20,250 households were selected and 20,127 women between the ages of 15 and 49 were interviewed. Among them, 18,895 were married women. The complete process of sample design and sample selection is shown in Figure 1.

### 2.3. Dependent Variable

The preliminary outcome of the study was the status of pregnancy intentions. Therefore, pregnancy intentions were considered dependent variables for this study that emerged from investigating whether women intended their current pregnancies. The BDHS tried to collect information about “whether a woman wanted a current pregnancy” and got three types of responses:

1. Then
2. Later
3. Not at all

To evaluate a woman's pregnancy intentions using BDHS data, we recoded these three responses as

1. “Then” for “Intended”; which code was zero (0)
2. “Later” and “Not at all” for “Unintended”; which code was one (1)

This method had been discussed by numerous authors in literature [7, 8]. In this study, we applied a machine learning approach to evaluate various algorithms' performance.

### 2.4. Explanatory Variables

A set of categorical explanatory variables were selected. According to various studies, fourteen explanatory variables were considered independent variables, namely, division (Barisal, Chittagong, Dhaka, Khulna, Mymensingh, Rajshahi, Rangpur, Sylhet) [8], sex of household head (Male, Female) [8], women's age group in years (15–19, 20–24, 25–29, 30–49) [19], wealth status (Poor, Middle, Rich) [20], women's educational level (No education, Primary education, Secondary and above) [19, 21], respondent's working status (Yes, No) [21], partner's age group (<25, 25–34, >34), partner's educational level (No education, Primary education, Secondary and above), intention of contraceptive use (Intended to use, Unintended to use) [8], age at first birth (Early, Not early, Don't know), age at first cohabitation (<18, ≥18) [8], number of living children (0, 1-2, 3+) [21], family size (<4, 4–6, >6) [8], and current residence with a partner (living with partner, staying elsewhere) [8].

### 2.5. Statistical Analysis

In this study, we conducted a simple descriptive analysis and bivariate analysis. We started with descriptive analysis to describe the frequency and percentage distribution. We used bivariate analysis to examine the association between pregnancy intention and selected independent variables. In the bivariate setting, we applied the independence test. For the independence test, we used the chi-square statistic, and it can be defined as

(1) $$\begin{array}{c} \chi^{2}=\sum \frac{{\left(O_{i}-E_{i}\right)}^{2}}{E_{i}};\;i=1,\ldots ,n, \end{array}$$

where *O*_*i*_ and *E*_*i*_ are the observed and expected frequency, respectively. The *χ*^2^ statistic asymptotically follows the *χ*^2^ distribution with the degrees of freedom (*r* − 1)(*c* − 1), where *r* is the number of categories for the independent variable and *c* is the number of categories for the dependent variable.

In a multivariable setup, we used six different supervised machine learning algorithms to predict the outcome variable and evaluate their performance in terms of model evaluation parameters.

In this study, we used six different popular ML algorithms:

1. Logistic regression
2. Random forest
3. Support vector machine
4. K-nearest neighbors
5. Naïve Bayes
6. Penalize regression (elastic net regression)

The following are some important considerations when choosing an algorithm.

The training data is smaller, so we have chosen highly interpretative algorithms named logistic regression, which have a low variance. Higher accuracy typically leads to a longer training time. We used naïve Bayes and logistic regression, which are easy to implement and quick to run. Since all attributes were categorical, so we require other algorithms that can handle high-dimensional and complex data structures. For that case, we have used random forest. Sometimes, a dataset may have a large number of irrelevant features. Besides, it can make training time unfeasibly long. The support vector machine is better suited in the case of data with broad feature space and lesser observations. That is why we have included that in our model. It is quite impossible to obtain a real-life dataset without a multicollinearity problem [22]. If the variables are intercorrelated, then parameter estimates have high variance and making the model unreliable. Elastic net regression is a combination of two convex penalty functions, such as ridge penalty and Least Absolute Shrinkage and Selection Operator (LASSO) penalty.

#### 2.5.1. Logistic Regression (LR)

Logistic regression (LR) is a “statistical learning” technique, which is a “supervised” machine learning (ML) method specifically used for “classification” tasks. It uses the maximum likelihood estimation procedure to estimate the parameters of interest. Let *X*_1_, *X*_2_,…, *X*_*p*_ be *p* number of regressors, which can be numerical variables or index variables that refer to the level of categorical variables, and *Y* is a binary variable, which has a Bernoulli distribution of the parameter *π*; then, the logistic regression model is

(2) $$\begin{array}{c} \log\left[\frac{\pi }{1-\pi }\right]=\beta_{0}+\beta_{1}X_{1}+\cdots +\beta_{p}X_{p}, \end{array}$$

where *β*_0_, *β*_1_,…, *β*_*p*_ are the unknown coefficients or parameters.

#### 2.5.2. Random Forest (RF)

Random forest is a classification method based on ensemble learning, and a large number of decision trees will be built during the training process, where the final output integrates the outcome class of individual decision trees [23].

#### 2.5.3. Support Vector Machine (SVM)

The support vector machine (SVM) is one of the most popular classification algorithms, which has a good way of transforming nonlinear data [24]. Pisner and Schnyer explained the classification strategy of SVM well [25]. The linear support vector machine model is used in the prediction research for mental health diseases [26], sentiment analysis [27], and so on.

#### 2.5.4. K-Nearest Neighbors (KNNs)

The K-nearest neighbors algorithm is also the simplest and one of the most widely used classification algorithms in machine learning algorithms. The KNN algorithm has confirmed the multiclass label classification problem and has good generalization ability [28]. The algorithm stores each accessible case and classifies new cases based on similarity measures.

#### 2.5.5. Naïve Bayes (NB)

The naïve Bayes (NB) classifier is a probabilistic classifier based on the assumption of strong (naïve) independence between the features of the Bayes theorem [29]. The naïve Bayes model is easy to construct without estimating complex repeat parameters, which makes it particularly effective in the treatment field. Although simple, naïve Bayes classifiers usually perform well and are widely used because they outperform more complex classification methods [30].

#### 2.5.6. Elastic Net Regression (ENR)

Penalized regression, also known as penalty regression, is a multivariate predictive model used for individual prediction or diagnosis checklist which is used to develop and validate risk model. Regularization is a technique that adds a penalty term to the objective function to avoid the overfitting of the data. This penalty controls the complexity of the model by shrinking the values of regression coefficients. There are various types of regularization techniques such as L1, L2, dropout, early stopping, and data augmentation are some of the most popular. LASSO regression uses the L1 regularization technique whereas ridge regression uses L2. Elastic net regression (ENR), another effective predictive model, combined both types of regularization [31].

### 2.6. Proposed Approach

First, we apply data preparation methods; for example, we exclude missing values from the data set and process them. In the case of a large amount of data, the best way is to randomly divide the entire data set into three parts: training set, validation set, and test set. We use the data from the training set to fit the model, the test set is used to estimate the prediction error of the model selection, and the test set is used to estimate the generalization error of the selected final model [32, 33]. Due to insufficient research data, the entire data set is divided into two parts: training and test. Here, 70% of the total sample taken randomly (called the training data set) is used to apply the ML algorithm and the remaining 30% of the total sample (called the test data set) is verified. We used 10-fold repeated cross-validation on the training set and evaluated the performance on the test set.

### 2.7. Model Evaluation: The Following Seven Evaluation Parameters Were Taken into Consideration

#### 2.7.1. Accuracy

For estimating the performance of predictive models, accuracy is the basis. It estimates the ratio of the correct estimate to the number of evaluated data points. It can be calculated as

(3) $$\begin{array}{c} \text{Accuracy}=\;\frac{\text{True Positive}+\text{True Negative}}{\text{True Positive}+\text{True Negative}+\text{False Positive}+\text{False Negative}}. \end{array}$$

#### 2.7.2. Sensitivity

Sensitivity measures how the model is mitigated to identify events in the positive class. It is also termed recall. Mathematically, sensitivity can be estimated as follows:

(4) $$\begin{array}{c} \text{Sensitivity}=\frac{\text{True Positive}}{\text{True Positive}+\text{False Negative}}. \end{array}$$

#### 2.7.3. Specificity

Specificity measures negative ratios to be accurately identified. This can also be presented in the form of a false positive rate. Mathematically, specificity can be estimated as follows:

(5) $$\begin{array}{c} \text{Specificity}=\frac{\text{True Negative}}{\text{True Negative}+\text{False Positive}}\text{.} \end{array}$$

#### 2.7.4. Positive Predictive Value

If we want to know how often a positive test delineates a true positive, positive predictive value helps us in this case. It is the proportion of positive results that comes from true positive and false positive. Mathematically, a positive predictive value can be estimated as

(6) $$\begin{array}{c} \text{Positive predictive value}=\frac{\text{True Positive}}{\text{True Positive}+\text{False Positive}}. \end{array}$$

#### 2.7.5. Negative Predictive Value

The negative predictive value is the proportion of negative results that comes from the result of true negative and false negative where a true negative is an event that makes a negative prediction and the results are also negative. This term is also denoted by specificity. On the other hand, a false negative is an event that makes a negative prediction but the result is positive. It is known as Type II error. A negative predictive value can be calculated as

(7) $$\begin{array}{c} \text{Negative predictive value}=\frac{\text{True Negative}}{\text{True Negative}+\text{False Negative}}. \end{array}$$

#### 2.7.6. Cohen's Kappa

Cohen's Kappa (*κ*) statistics is a good measure for dealing with multiclass and unbalanced classification problems. It is a ratio between the predicted and the actual classifications in a data set and an understanding of the actual taxonomy. The range of Cohen's Kappa is ≤1. According to Landis and Koch, when Cohen's Kappa value <0, it indicates no agreement, 0 to 0.20 slight, 0.21 to 0.40 fair, 0.41 to 0.60 moderate, 0.61 to 0.80 substantial, and 0.81 to 1 almost perfect agreement [34].

#### 2.7.7. Area under the ROC Curve

The area under the ROC curve is a performance measurement for classification problems in various threshold configurations. ROC is a probability curve and AUC represents the degree or measure of separability. It tells how much the model is capable of distinguishing between classes. The higher the AUC, the better the model is at predicting 0 s as 0 s and 1 s as 1 s [35].

### 2.8. Analytical Tools

For data management and analysis, the SPSS (Statistical Package for Social Science) 25 version and R-programming version 4.0.0 were used.

## 3. Results

Table 1 depicts the background characteristics of the women participating in the study. The highest number of respondents was from Chittagong (15.4%) and Dhaka (15.3%) divisions. Almost all respondents (89%) were from a male-headed household. Most participants (34.4%) were between 20 and 24 years of age. The majority of the participants were from poor and rich wealth statuses (approximately, 40%, each). Only 18.8% of respondents belong to middle-class families. More than two-thirds (69%) of the respondents had completed secondary or higher education. The proportion of unemployed women is 67.2%. It was found that half of the women's husbands (51.6%) were between 25 and 34 years of age, whereas 54.2% of them had completed secondary or higher education. Almost all women (98.6%) plan to use contraceptive methods. More than two halves (67.1%) of the women of the first cohabitation were found to be less than 18 years old, and 50.5% of the women had 1-2 children. 47.9% of the respondents had a family of 4 to 6 members. Most of the women (82%) were living with their partners.

The prevalence of unintended pregnancy and the background characteristics of the selected covariates are shown in Table 2. From the *χ*^2^ test, all the covariates were found significantly associated with unintended pregnancy (*P* < 0.001; *P* < 0.01; *P* < 0.05). The percentage of women with an unintended pregnancy is found to be higher for the Sylhet division (33.8%), women living in a male-headed household (26.5%), women in the age group 30 to 49 (35.5%), women with poor wealth status (29.7%), women without education (43.8%), employed women (29.2%), women with husband's age more than or equal 35 years (30%) and without education (41.5%), women with contraceptive intention (25.2%), women with early birth age (38%), first cohabitation at less than 18 years of age (28.4%), women having 3 or more children (56.7%), women with 4 to 6 family members (28.3%), and women living with their partner (26.6%).

It should be noted that multicollinearity is one of the assumptions to implement any regression model. The existence of multicollinearity will reduce the accuracy of the estimated coefficients. For this reason, we checked the multicollinearity before performing the selected supervised models. We observed that there was moderate multicollinearity present in this analysis. However, moderate multicollinearity may not be a big problem [22].

In this study, six different ML algorithms were applied to classify the current pregnant women as unintended pregnant and intended pregnant in the test data set. Performance parameters (such as accuracy, sensitivity, specificity, and AUC value) were used to compare the predictive performance of these algorithms. In addition, Cohen's Kappa statistical information is used to determine the discriminative accuracy of the algorithm. The prediction results with performance parameters for each algorithm are shown in Table 3 and Figure 2.

In Table 3, we see that the test data accuracy of the logistic regression (LR) classifier is 79.29%, which means that the algorithm is 79.29% correct for the prediction. The sensitivity and specificity of the logistic regression were 29.76% and 95.67%, respectively.

In this study, a pair model tuning parameter was used for the best performance of the random forest (RF) classifier. Although there are many parameters for RF, we chose two parameters that provide the best effect on the final accuracy. Those parameters are the “number of variables randomly sampled” (denoted by “mtry”) and “number of trees to grow” (denoted by “*n*tree”). For the study, we found the best mtry is 2 and the best ntree is 500 through 10-fold cross-validation. Therefore, we get an accuracy of 77.81%, sensitivity of 11.91%, and specificity of 99.61% for RF.

In the case of a support vector machine (SVM), our model tuning parameter is the cost/capacity parameter which is generally chosen via cross-validation and determines the number and severity of violations to the hyperplane that data will tolerate. In this study, the value of *C* was 0.1 and the final accuracy was 76.92% with 21.43% and 95.28% sensitivity and specificity, respectively.

Using k-nearest neighbor (KNN), the accuracy in the test data set was seen as 77.22% with sensitivity and specificity of 10.71% and 99.21%, respectively. Here, the number of nearest neighbors was 17.

According to the test observation results, the naïve Bayes method (NB) showed 78% accuracy in predicting unintended pregnancy, with a sensitivity of 12.62% and a specificity of 99.83%.

Finally, we look for the elastic net regression model (ENR), which is the combination of two popular penalties (ridge regression alpha (*α*) = 0 and LASSO regression alpha (*α*) = 1). Here, the two model parameters are lambda (*λ*) and alpha (*α*). In this study, alpha (*α*) has a value of 0.594, lambda (*λ*) has a value of 0.006, and we get an accuracy of 77.51%, sensitivity of 17.86%, and specificity of 97.24%.

Among the six classifiers, we obtain the best performance of LR with an accuracy of 79.29%. Although accuracy is a parameter for evaluating performance, we estimate model performance based on the ROC (receptor performance) curve and the AUC (area under the ROC curve) value. Because the overall accuracy is based on a cut point, while ROC curve tries all the cut point and plot the sensitivity and 1− specificity. If we try to interpret the model performance depending on accuracy, we only consider a particular cut point. But overall accuracy varies with different cut points, which are taken into account when drawing the ROC curve. Furthermore, AUC is the measure of separability that indicates the model's capability in distinguishing between classes. Thus, in practice, the ROC curve and the AUC can give us more accurate information than accuracy.

Depending on the AUC value (Figure 2), we can see that ENR produces a great distinction between intended and unintended pregnancy among all classifiers; i.e., it gives a more accurate prediction (approximately 75%) than others.

## 4. Discussion

To the best of our knowledge, this is the first study to predict unintended pregnancy using machine learning classifiers among women in Bangladesh. The key objective of this research is to predict unwanted pregnancies between married women in Bangladesh. Six well-known machine learning algorithms are applied to meet the research goals, such as logistic regression, random forest, k-nearest neighbor, support vector machine, naïve Bayes, and elastic net regression. We trained all models based on 10-fold cross-validation on the training data set and evaluated performance on the test data set. By using the *χ*^2^ test, all covariates are significantly related to the outcome variables.

The prediction performance of these six machine learning algorithms is compared based on the curve value area. Many authors have made comparisons based on accuracy [16]. However, several authors have shown that AUC is a better method than accuracy, in both experience and form [36]. According to the ROC curve area, the best result has been obtained by the elastic net regression algorithm. The AUC of the elastic net regression algorithm is about 74%. The variance-bias trade-off, multicollinearity, feature selection, and easier interpretation of the output are all factors that are taken into account when developing ENR models. That is why ENR outperforms other current models for our datasets due to all of these properties [37]. However, in the study in Missouri, the researchers found that random forest performed better than other machine learning techniques in predicting unintended birth and pregnancy [38]. Furthermore, they did not apply the elastic net regression algorithm in their analysis. On the contrary, the neural network produced the highest area under the ROC curve compared to other machine learning algorithms included in their studies [39, 40]. To predict unwanted pregnancy among women aged 35 or more in Iran, Nouhjah and Kalhori applied artificial neural networks and revealed that the area under the curve for artificial neural was 0.67 [41].

In the different settings, Huang et al. suggested that the endometrial immunology panel had the largest area under the curve (AUC = 0.766) in terms of biochemical pregnancy prediction [42]. A systematic review of 127 individual studies conducted by researchers [43] observed that machine learning and artificial intelligence technologies, particularly recent deep learning (DL) methods (*n* = 13), are being used to improve pregnancy outcomes. Islam and his team members proposed that stacking classification (SC) produces the highest f1 score when predicting the mode of childbirth when compared to the other machine learning techniques included in their analysis [44]. Based on various performance parameters, a new stack ensemble (SE) classifier is proposed, which outperforms the compared other classifiers for predicting stillbirth [45]. In a different context, the Extreme Randomized Forest approach had the best accuracy and area under the curve when it came to predicting pregnant women with depression symptoms [46].

This research has some limitations. When the predictive model is built using DHS cross-sectional data, it cannot access additional information about other related factors. Combining these factors may increase predictive accuracy and AUC. However, this study proves that machine learning algorithms can predict unwanted pregnancies based on general risk factors that can help in the development of interventions to improve planned pregnancies and family planning among married couples in Bangladesh.

## 5. Conclusions

In this study, we compared six machine learning algorithms to predict whether a woman might become pregnant unexpectedly. Among the algorithms considered, the elastic net regression algorithm showed the best results and the most accurate classification for predicting unwanted pregnancy among Bangladeshi women. Additionally, our findings would be valuable for identifying women at risk of unintended pregnancy. Therefore, plans and guidelines should be developed to improve the use of contraceptive methods and strengthen marriage communication related to pregnancy.

## Figures and Tables

**Figure 1:** Study population and sample selection procedure for this study.

**Figure 2:** Performance evaluation of various classification techniques using ROC curve.

**Table 1:** Background characteristics of the study participants.

Variables	Frequency (*n = *1129)	Percent (%)
*Division*		
Barisal	114	10.1
Chittagong	174	15.4
Dhaka	173	15.3
Khulna	121	10.7
Mymensingh	146	12.9
Rajshahi	121	10.7
Rangpur	126	11.2
Sylhet	154	13.6
*Sex of Household Head*		
Male	1001	88.7
Female	128	11.3
*Woman's Age Group (in years)*		
15-19	314	27.8
20-24	388	34.4
25-29	255	22.6
30-49	172	15.2
*Wealth Status*		
Poor	458	40.6
Middle	212	18.8
Rich	459	40.7
*Education Status*		
No education	48	4.3
Primary education	303	26.8
Secondary and above	778	68.9
*Respondent Occupation*		
Yes	370	32.8
No	759	67.2
*Husband Age*		
≤24	166	14.7
25-34	582	51.6
≥35	381	33.7
*Husband's Education Status*		
No education	142	12.6
Primary education	375	33.2
Secondary and above	612	54.2
*Contraceptive Intention*		
Intended to use	1113	98.6
Unintended to use	16	1.4
*Age at first birth*		
Early	309	27.4
Not early	376	33.3
Don't Know	444	39.3
*Age at First Cohabitation*		
<18	758	67.1
≥18	371	32.9
*Number of Children*		
0	469	41.5
1-2	570	50.5
3+	90	8.0
*Family Size*		
4<4	255	22.6
4-6	541	47.9
>6	333	29.5
*Partner Residence*		
Living with partner	925	81.9
Staying elsewhere	204	18.1
*Involuntary Pregnancies*		
Intended	847	75.0
Unintended	282	25.0

**Table 2:** Percentage distribution and association between selected covariates and women's pregnancy intentions in Bangladesh.

Variables	Current Pregnancy Intention		*χ* ^2^value	*p* value
	Intended (*n* = 847)	Unintended (*n* = 282)		
*Division*			24.91	<0.001
Barisal	75.4	24.6		
Chittagong	83.9	16.1		
Dhaka	75.1	24.9		
Khulna	83.5	16.5		
Mymensingh	77.4	22.6		
Rajshahi	70.2	29.8		
Rangpur	66.7	33.3		
Sylhet	66.2	33.8		
*Sex of Household Head*			10.54	<0.001
Male	73.5	26.5		
Female	86.7	13.3		
*Women's age group (in years)*			13.06	0.005
15-19	79.0	21.0		
20-24	76.3	23.7		
25-29	75.3	24.7		
30-49	64.5	35.5		
*Wealth status*			12.73	0.002
Poor	70.3	29.7		
Middle	73.6	26.4		
Rich	80.4	19.6		
*Education status*			22.20	<0.001
No education	56.3	43.8		
Primary education	68.3	31.7		
Secondary and above	78.8	21.2		
*Respondent occupation*			5.21	0.01
Yes	70.8	29.2		
No	77.1	22.9		
*Husband age*			7.57	0.02
≤24	78.3	21.7		
25-34	77.3	22.7		
≥35	70.1	29.9		
*Husband education status*			39.65	<0.001
No education	58.5	41.5		
Primary education	70.4	29.6		
Secondary and above	81.7	18.3		
*Contraceptive intention*			4.04	0.04
Intended to use	74.8	25.2		
Unintended to use	93.8	6.3		
*Age at first birth*			72.32	<0.001
Early	62.1	37.9		
Not early	70.2	29.8		
Don't Know	88.1	11.9		
*Age at first cohabitation*			14.12	<0.001
<18	71.6	28.4		
≥18	81.9	18.1		
*Number of children*			102.76	<0.001
0	88.3	11.7		
1-2	69.1	30.9		
3+	43.3	56.7		
*Family size*			9.00	0.01
<4	81.6	18.4		
4-6	71.7	28.3		
>6	75.4	24.6		
*Partner residence*			7.14	0.004
Living with partner	73.4	26.6		
Staying elsewhere	82.4	17.6		

**Table 3:** Performance indicators of all five machine learning algorithms to predict pregnancy intention among married women in Bangladesh.

	LR	RF	SVM	KNN	NB	ENR
*Training data set*						
Accuracy (%)	76.99	78.00	75.98	76.11	77.22	77.12
95% CI	(73.90, 79.88)	(74.95, 80.84)	(72.85, 78.92)	(72.98, 79.04)	(72.37, 81.58)	(74.03, 80.00)
*κ*	0.2319	0.1830	0.1629	0.1147	0.1302	0.1600
Sensitivity (%)	23.74	13.64	16.67	10.10	10.52	13.13
Specificity (%)	94.77	99.49	95.78	98.15	99.61	98.48
PPV (%)	60.26	90.00	56.90	64.52	88.89	74.29
NPV (%)	78.82	77.53	77.49	76.58	76.90	77.25

*Testing data set*						
Accuracy (%)	79.29	77.81	76.92	77.22	78.00	77.51
95% CI	(74.57, 83.48)	(73.00, 82.13)	(72.06, 81.31)	(72.37, 81.58)	(74.95, 80.84)	(72.68, 81.86)
*κ*	0.3144	0.1623	0.2128	0.1400	0.1753	0.2005
Sensitivity (%)	29.76	11.91	21.43	10.71	12.62	17.86
Specificity (%)	95.67	99.61	95.28	99.21	99.83	97.24
PPV (%)	69.44	90.91	60.00	81.82	96.15	68.18
NPV (%)	80.46	77.37	78.57	77.06	77.39	78.16

PPV = positive predictive value, NPV = negative predictive value.

## Data Availability

In this study, we used data from Bangladesh Demographic Health Survey (BDHS), 2017-18, which is available from https://dhsprogram.com/data/available-datasets.cfm.
